The article "Cuproptosis-Related Genes CDK1 and COA6 Involved in the Prognosis Prediction of Liver Hepatocellular Carcinoma" was retracted in 2023. Reasons: signs of a paper mill; compromised peer review; unreliable results or conclusions.

# Cuproptosis-Related Genes CDK1 and COA6 Involved in the Prognosis Prediction of Liver Hepatocellular Carcinoma

**DOI:** 10.1155/2023/5552798

**Published:** 2023-05-11

**Authors:** Sanfeng Han, Tao Ye, Yuqin Mao, Bo Hu, Chen Wang

**Affiliations:** ^1^Central Laboratory, Institute of Fudan-Minhang Academic Health System, Minhang Hospital, Fudan University, China; ^2^Department of Oncology, Minhang Hospital, Fudan University, China; ^3^Key Laboratory of Whole-Period Monitoring and Precise Intervention of Digestive Cancer (SMHC), Minhang Hospital & AHS, Fudan University, China; ^4^Center for Traditional Chinese Medicine and Gut Microbiota, Minhang Hospital, Fudan University, 201199 Shanghai, China

## Abstract

**Background:**

Liver hepatocellular carcinoma (LIHC) is the most frequently seen type of primary liver cancer. Cuproptosis is a novel form of cell death highly associated with mitochondrial metabolism. However, the clinical impact and pertinent mechanism of cuproptosis genes in LIHC remain largely unknown.

**Methods:**

From public databases, we systematically assessed common genes from LIHC differentially expressed genes (DEGs) and cuproptosis-related genes using bioinformatics analysis. These common genes were then analyzed by enrichment analysis, mutation analysis, risk score model, and others to find candidate hub genes related to LIHC and cuproptosis. Next, hub genes were determined by expression, clinical factors, immunoassay, and prognostic nomogram.

**Results:**

Based on 129 cuproptosis-related genes and 3492 LIHC DEGs, we totally identified 21 downregulated and 18 upregulated common genes, and they were enriched in pathways, such as zinc ion homeostasis and oxidative phosphorylation. In the mutation analysis, missense mutation was the most common type in LIHC patients, and the common gene F5 had the highest mutation frequency. After LASSO-Cox regression analysis and prognostic analysis, CDK1, ABCB6, LCAT, and COA6 were identified as prognostic signature genes. Among them, ABCB6 and LCAT were lowly expressed in tumors, and CDK1 and COA6 were highly expressed in tumors. In addition, ABCB6 and LCAT were negatively correlated with 6 kinds of immune cells, while CDK1 and COA6 were positively correlated with them. CDK1 and COA6 were identified as hub genes related to LIHC by Cox regression analysis and prognostic nomogram.

**Conclusion:**

CDK1 and COA6 are two oncogenes in LIHC, which are involved in the molecular mechanism of cuproptosis and LIHC. Besides, CDK1 and COA6 can positively regulate the expressions of immune cells in LIHC. In clinical practice, they can be used as immunotherapeutic targets and prognostic predictors in LIHC, which sheds new light on the scientific fields of cuproptosis and LIHC.

## 1. Background

The second most common cause of cancer-related death globally is primary liver cancer [1]. According to histological types, primary liver cancer is divided into four categories: fibrous liver cancer, intrahepatic cholangiocarcinoma, hepatocellular cholangiocarcinoma, and liver hepatocellular carcinoma (LIHC) [2, 3]. 90% of primary liver cancer cases are caused by LIHC, and this global problem kills more than 700,000 people every year [4, 5]. Due to the late diagnosis, rapid tumor growth, and early postoperative recurrence of LIHC, clinical treatment methods are limited, including partial keratectomy, hepatic chemotherapy, hepatic radiofrequency ablation, transarterial hepatic chemoembolization, liver transplantation, and molecularly targeted therapy [6]. The efficacy of this treatment modality remains limited. Common factors contributing to this are the lack of timely diagnosis and the high rate of recurrence in most LIHC patients [7]. Therefore, it is an urgent need to explore the mechanisms of LIHC and identify effective biomarkers for early detection.

Since copper's homeostasis may become dysregulated, it can lead to cytotoxicity [8]. Copper is a crucial trace metal involved in many biological processes [9]. Recent studies have shown that when compared to healthy individuals, cancer patients have considerably higher blood and tumor copper levels, suggesting that changes in intracellular copper levels may have an impact on the onset and progression of cancer [10, 11]. The use of copper ionophores and copper chelators in anticancer treatment is based on this process. Tsvetkov et al. describe a copper-dependent cell death (called cuproptosis, a nonapoptotic cell death pathway) in recent research published in *Science*. It has been shown that the fatty acrylate part of the tricarboxylic acid (TCA) cycle is directly bound by copper. These copper-bound fatty acrylate mitochondrial proteins aggregate, leading to the loss of Fe-S cluster proteins, which in turn results in phototoxic stress and a particular type of cell death [12]. In recent years, increasing evidence has confirmed the importance of cuproptosis in regulating tumor cell proliferation, growth, and metastasis. For example, Bian et al. showed that a cuproptosis-associated gene signature could serve as a potential prognostic predictor in patients with clear cell renal cell carcinoma, which might provide new insights into cancer therapy [13]. In addition, studies by Lv et al. demonstrated the prognostic value of cuproptosis-related genes in melanoma, especially LIPT1, and revealed the correlation between LIPT1 expression and immune infiltration in melanoma [14]. These findings all illustrate the important roles of cuproptosis genes in the treatment and prognosis of cancers.

In recent years, studies related to cuproptosis-related genes (CRGs) in LIHC patients have been reported [15]. However, in this field, there are few reports on the potential biomarkers with clinical practice in LIHC patients. Therefore, we intend to comprehensively investigate the potential mechanism by analyzing CRGs and LIHC-related differentially expressed genes (DEGs) in LIHC. Our research will provide valuable experience in the field of cuproptosis and LIHC and lay the foundation for the clinical application of CRGs in LIHC.

## 2. Materials and Methods

### 2.1. The Cancer Genome Atlas (TCGA) Database

The TCGA database (https://portal.gdc.com) provided the clinical, transcriptome, and gene mutation data for the LIHC dataset. Using the “normalize between arrays” function of the “limma” R package (version 3.40.2), the data obtained from the TCGA and GTEx databases were rectified and normalized.

### 2.2. Differential Expression Analysis and Validation

We screened TCGA-LIHC DEGs under |log2(fold change)| > 1 and *P* < 0.05. Subsequently, Venn diagrams of CRGs (from gene set enrichment analysis, GSEA website) and TCGA-LIHC DEGs were generated using the Venn diagram package in R software (R software, version 3.5.1). Also, we identified up- and downregulated properties of common genes. The Database for Annotation, Visualization and Integrated Discovery (DAVID) then carried out Gene Ontology (GO) and Kyoto Encyclopedia of Genes and Genomes (KEGG) pathway enrichment analyses on common genes, which were both visualized using the “ggplot2” package of the R (version 3.40.2) project (*P* < 0.05). The examination of GO enrichment comprised cellular components (CC), biological process (BP), and molecular function (MF).

### 2.3. Gene Set Cancer Analysis (GSCA)

The CNV (copy number variation) and SNV (single nucleotide variation) of the mutant gene were determined by the GSCA database (http://bioinfo.life.hust.edu.cn/GSCA/) [16]. To comprehensively study somatic mutations in LIHC patients in the TCGA database, somatic mutations in LIHC patients were downloaded and visualized by the maftools package in R software (R software, version 3.5.1). Horizontal histograms showed that LIHC patients had a higher frequency of gene mutations.

### 2.4. LASSO (Least Absolute Shrinkage and Selection Operator) Regression Analysis

The “glmnet” package of the R programming language (v4.0.3 version) was used to use LASSO regression analysis to create a polygenic signal with LIHC for predicting the prognosis of LIHC. Tenfold cross-validation was used to extract the ideal value from the smallest partial likelihood deviation to increase the accuracy and objectivity of the analytical results. TCGA-LIHC patients were divided into high-risk and low-risk groups based on the median risk score as a cutoff. Survival differences between the above two groups were compared by the Kaplan-Meier survival analysis. Time-dependent receiver operating characteristic (ROC) plots were drawn to determine whether risk scores accurately predicted survival status.

### 2.5. The Tumor Immunity Estimation Resource (TIMER)

The Wilcox tests were adopted to compare the expression levels of the prognostic genes from the risk score model in LIHC tumors and T, N, and M stages. The TIMER online interface is user-friendly and may be used to research the molecular characterization of tumor-immune interactions. The correlation of the 4 prognostic genes with the 6 immune cells was analyzed by the correlation module in TIMER.

### 2.6. Construction and Validation of Gene Prediction Nomogram

To assess the predictive power and several clinical factors, such as T and M stage and age, univariate and multivariate Cox proportional hazards regression analyses were conducted on prognostic genes to filter all the independent prognostic factors. Then, a composite nomogram was constructed to predict the probability of 1-, 3-, and 5-year overall survival (OS) by “rms” package of the R software (R software, version 3.5.1). Additionally, nomogram predictions and observations could be compared by calibration curves.

## 3. Results

### 3.1. 39 Common Genes Were Screened from TCGA-LIHC DEGs and CRGs

In total, we identified 2558 upregulated and 934 downregulated DEGs (Figure 1(a)).  Figure 1(b) is a Venn diagram of 129 CRGs and 3492 TCGA-LIHC DEGs, and 39 overlapping genes were determined.  Figure 1(c) is the up- and downregulated properties of 39 overlapping genes, including 21 down- and 18 upregulated genes. These genes were enriched in zinc ion homeostasis and response to zinc ion (BP, Figure 1(d)); Golgi-associated vesicle and multivesicular bodies, among others (CC, Figure 1(e)); and phosphatidylcholine-sterol O-acyltransferase activator activity and apolipoprotein A-I binding, among others (MF, Figure 1(f)). The enriched KEGG pathways included oxidative phosphorylation and progesterone-mediated oocyte maturation, among others (Figure 1(g)).

### 3.2. The Mutational Landscape of Somatic Mutations in the 39 Genes

Next, we performed a genetic variation analysis on the above 39 genes, including CNVs and SNVs, using the GSCA database. We analyzed the CNV percentages of 39 genes in LIHC and found that the LOXL2 gene had the highest percentage of CNVs (Figure 2(a)). As shown in Figure 2(b), the percentage of SNVs for 33 genes in LIHC was demonstrated, and the results showed that the F5 gene had the highest SNV. Missense mutations were the most prevalent kind of mutation in LIHC patients. Single nucleotide polymorphisms (SNPs) were the main type of mutational variation, with *C* > *T* occupying an absolute position. The median mutational variation per sample was 1, and each color box represented a mutation. In addition, the top 10 mutated genes were F5 (18%), APP (13%), LOXL4 (9%), LCAT (7%), DAXX (7%), AQP1 (7%), STEAP4 (4%), STEAP3 (4%), APOA4 (4%), and ABCB6 (4%) (Figure 2(c)). Horizontal histograms demonstrated the top 10 mutated genes with the highest mutation frequency in LIHC patients (*n* = 45; Figure 2(d)).

### 3.3. Four Prognostic Genes Were Identified from the Risk Score Model

Four prognostic genes (CDK1, ABCB6, LCAT, and COA6) were finally identified in the LASSO analysis (Figures 3(a) and 3(b)). By the median risk score, LIHC patients were separated into low-risk and high-risk groups (*n* = 181).  Figure 3(c) shows the survival status of all patients and the expression heatmap of the 4 prognostic genes. The Kaplan-Meier curve analysis showed that high-risk patients were related to poorer disease-specific survival (DSS) compared with low-risk patients (Figure 3(d)). Furthermore, ROC curve analysis showed that the area under the ROC curve (AUC) of the predictive model at 1, 3, and 5 years was 0.833, 0.777, and 0.622 in the training set, respectively (Figure 3(e)).

### 3.4. The Clinical Factor Analysis and Immunoassay on the 4 Prognostic Genes

The level of ABCB6 in tumor tissues was lower than in the other group (Figure 4(a)). Second, the expression of ABCB6 was lower in each subgroup of T, N, and M phases than in normal tissues (Figures 4(b)–4(d)). In contrast, the levels of CDK1 and COA6 were higher in tumor tissues and clinicopathological stages than in normal tissues (Figures 4(e)–4(l)). Then, the levels of LCAT in tumor tissues and clinicopathological stages were lower (Figures 4(m)–4(p)). The levels of ABCB6 and LCAT were negatively related to 6 immune cells (T cell CD4, B cell, T cell CD8, macrophage, neutrophil, and DC (Figures 5(a) and 5(d), *r* < 0). However, the expressions of CDK1 and COA6 were positively correlated with the 6 immune cells (Figures 5(b) and 5(c), *r* > 0).

### 3.5. CDK1 and COA6 Were the Hub Genes Involved in the Molecular Mechanism of Cuproptosis and LIHC

After the Cox analysis, we found that CDK1, COA6, and pT-stage were independent prognostic variables for LIHC (Figure 6(a)). Then, we constructed a composite nomogram integrating CDK1, COA6, and pT-stage to predict 1-, 3-, and 5-year OS in LIHC patients (Figure 6(b)). The gene prognosis nomogram's anticipated outcomes and actual results were in good agreement, as seen by the calibration plot for patient survival prediction (Figure 6(c)).

## 4. Discussion

Studies have shown that copper, platinum, and iron extensively studied in the development of drug delivery systems show a promising promise in a range of anticancer uses [17]. A variety of copper ionophore drugs such as elesclomol (ES), disulfiram, and NSC319726 can cause cell death [12]. This copper-induced cell death is a new type of death defined as cuproptosis, different from other programmed cell death [18]. Mutations that lead to copper excess can have serious consequences [19]. Nonetheless, it is possible to regulate intracellular copper levels in a range to destroy tumor cells in a targeted manner [20]. Cuproptosis, an untraditional cell death mechanism involving protein fatty acylation in the TCA cycle, may indicate new insights into the use of copper toxicity in tumor therapy [21]. The discovery of cuproptosis has opened up a refreshing pathway of cell death and gives a fresh approach to cancer treatment by fully using copper's pathophysiological effects [22]. Therefore, it is of much importance to explore the roles and functions of CRGs for the diagnosis, prevention, and treatment of LIHC. To our knowledge, no prior research has focused on the relationship between CRGs and LIHC growth. Most CRGs are strongly related to prognosis and immunity and differently expressed in tumor and normal tissues; this finding suggests that cuproptosis genes may have therapeutic significance in predicting LIHC prognosis.

Herein, we investigated the common genes from LIHC DEGs and CRGs and examined the functions of common genes in LIHC. From the pathway of common gene enrichment, it can be seen that common genes are mainly enriched in the homeostasis and response of metal ions in BP, like responses to copper ions, cellular transition metal ion homeostasis, cellular responses to cadmium ions, cellular responses to zinc ions, and zinc ion homeostasis. Furthermore, the enriched terms in CC were mostly organelle membranes and organelle lumen, including the binding membrane of organelles, endoplasmic reticulum lumen, mitochondrial envelope, and Golgi-related vesicles. Similarly, the enriched terms of common genes in MF included transition metal ion binding, copper ion binding, and cuprous ion binding. Overall, these genes are associated with copper ions as well as organelles. Studies by Li et al. show that copper homeostasis is tightly controlled in prokaryotes and eukaryotes, mostly by limiting the overabundance of copper ions in cells, which endangers cell viability [23]. In the enrichment analysis of KEGG, the enriched pathways of common genes included p53 signaling pathway and so on. One of the most well-known tumor suppressors is the protein p53 [24]. As a cell cycle checkpoint, p53 can identify cells with aberrant mutations, pause the cell cycle, reduce cell proliferation, and trigger apoptosis [25, 26]. Studies by Li et al. showed that the tumor suppressor gene p53 could significantly reduce the promoting effect of JMJD2D on the development of liver cancer cells [27]. This conclusion is consistent with the above research theory.

Next, evidence from mutation profiling indicated that 75.56% of LIHC patients harbored different types of mutations. The majority of the mutations in these affected genes in LIHC patients were missense mutations, with F5 having the greatest mutation frequency (18%). A significant number of missense mutations may change the genetic code by changing the structure and function of proteins, which raises the possibility that they play a part in the pathogenesis of LIHC. When compared to other SNV classes, *C* > *T* was the most common DNA base substitution in LIHC patients and SNP was the most common mutant variant type. Next, we established a risk model for common genes and screened out 4 prognostic genes. In expression analysis, two of the prognostic genes were LIHC proto-oncogenes (CDK1 and COA6), and two prognostic genes were LIHC tumor suppressor genes (ABCB6 and LCAT). Further immunoassay of prognostic genes showed that the levels of CDK1 and COA6 were positively related to T cell CD4, B cell, T cell CD8, macrophage, neutrophil, and DC, while the expressions of ABCB6 and LCAT are negatively related to them.

Further, CDK1, COA6, and pT-stage could be reliable prognostic variables for LIHC. A family of kinases known as CDK (cyclin-dependent kinase) is heavily engaged in controlling the cell cycle [28, 29]. The interaction between CDKs, their regulatory subunits, and CDK inhibitors regulates the transitions between cell cycle stages [30]. By interacting with cyclin B, CDK1 controls the G2-M transition and makes it easier to enter mitosis [31]. The coordinated entrance into mitosis is altered by CDK1 overexpression and depletion, and this can have an impact on the length of the G2-M arrest [32]. Ying et al. showed that CDK1 was overexpressed in endometriosis endometrial carcinoma based on experimental findings. Cells from endometrial carcinoma that had CDK1 activity inhibited underwent apoptosis and had a G2/M arrest, while also inhibiting endometrial cancer growth in a xenograft model [33]. COA6 (cytochrome c oxidase assembly factor 6) encodes a member of the 6B family of cytochrome c oxidase subunits [34]. Pacheu-Grau et al. suggest that hypertrophic cardiomyopathy is linked to the loss of COA6 function [35]. For copper to be inserted into the Cu_A_ center, the metal partners SCO1 and SCO2 must be present in combination with COA6. That means, COA6 can act as a copper metal chaperone thiol reductase, which is closely related to the mitochondrial respiratory chain [36].

In summary, this study systematically analyzes the common genes of LIHC and CRGs, and after a series of bioinformatics analyses, two oncogenes CDK1 and COA6 are obtained. Our analysis shows that the expressions of CDK1 and COA6 are upregulated in LIHC clinical tumor tissue samples with a good diagnostic value in LIHC. Thus, it is concluded that CDK1 and COA6 as two CRG oncogenes may be promising indicators for LIHC prognosis, which reveals the molecular mechanism between CRGs and LIHC and also provides new directions for LIHC clinical practice. However, further experimental studies are still needed to determine the specific mechanism of action.

## Figures and Tables

**Figure 1:** Identification of LIHC DEGs and acquisition of 39 common genes. (a) Volcano plot of DEGs in LIHC and normal tissue. Red represents upregulated DEGs, and green represents downregulated DEGs. The top ten upregulated DEGs were GPC3, AKR1B10, MDK, PLVAP, POLR2F, LYNX1, CXCL10, UBE2C, LYZ, and NQO1. The top ten downregulated DEGs included SAA4, APOC4, SERPINA3, A1BG, ITIH4, APOC2, ARL6IP4, RPL17, RPS10, and DDT. (b) Venn diagram of DEGs and CRGs. A total of 39 overlapping genes were screened out. (c) Histogram of 21 downregulated overlapping genes and 18 upregulated overlapping genes. Red ones represent upregulated overlapping genes, and blue ones represent downregulated overlapping genes. (d–f) Top ten BP, CC, and MF terms for 39 common genes. This graph is a combination of the Sankey graph and bubble graph; the larger the bubble, the more genes are enriched in this pathway. (g) Top 10 KEGG pathways of 39 common genes.

**Figure 2:** The mutational landscape of somatic mutations in the 39 genes. (a) Pie chart of CNV percentages for 39 overlapping genes in LIHC. (b) Heatmap of SNV percentages for 33 mutated genes in LIHC. (c) Cohort summary plot showing the distribution of variants by type, variant class, and SNV category. Missense mutations are the main mutation type. (d) Waterfall plots are used to display mutation data for each gene in each sample. The various mutation types are represented by different colors and specific annotations at the bottom of the waterfall chart.

**Figure 3:** Four prognostic genes were identified from the risk score model. (a) LASSO-Cox model fitting procedure. Each curve represents a gene. Plot the trend of each coefficient against the *L*1 norm as *λ* varies. The *L*1 norm is the total absolute value of the nonzero coefficients. (b) *λ* is selected by 10-fold cross-validation. (c) Risk score curves, patient survival, and heatmaps depicting the expression patterns of the four prognostic genes. (d) Difference in survival between high-risk and low-risk patients. Survival was poorer in the high-risk patient group. (e) Time-dependent ROC curve analysis of 1-, 3-, and 5-year overall survival predictions.

**Figure 4:** Clinical features of LIHC and prognostic genes expression. (a–d) ABCB6 expression in LIHC and T, N, and M stages. The yellow boxplot represents the tumor group, and the green boxplot represents the normal group. The significance of two groups of samples was tested by the Wilcox test, and the significance of the three groups of samples was tested by the Kruskal-Wallis test. (e–h) CDK1 expression in LIHC and T, N, and M stages. (i–l) COA6 expression in LIHC and T, N, and M stages. (m–p) LCAT expression in LIHC and T, N, and M stages. ^∗^*P* < 0.05, ^∗∗^*P* < 0.01, ^∗∗∗^*P* < 0.001, and ^∗∗∗∗^*P* < 0.0001. ns means not significant.

**Figure 5:** Immune correlation analysis on the 4 prognostic genes. (a) Immune correlation of ABCB6 with 6 immune cells. *r* < 0 means that the gene is negatively correlated with immune cells, and *r* > 0 means that the gene is positively correlated with immune cells. (b) Immune correlation of COA6 with 6 immune cells. (c) Immune correlation of CDK1 with 6 immune cells. (d) Immune correlation of LCAT with 6 immune cells.

**Figure 6:** Determination of independent prognostic parameters and construction of gene-based nomogram models. (a) Forest plots of univariate and multivariate Cox regression analyses of prognostic genes and clinical characteristics. (b) Nomogram of independent prognostic variables. C − index = 0.798; *P* < 0.001. (c) Nomogram calibration plots for the consistency check between 1-, 3-, and 5-year OS predictions and actual outcomes.

## Data Availability

The datasets used and/or analyzed during the current study are available from the corresponding authors on reasonable request.
